# A Novel Ensemble-Based Technique for the Preemptive Diagnosis of Rheumatoid Arthritis Disease in the Eastern Province of Saudi Arabia Using Clinical Data

**DOI:** 10.1155/2022/2339546

**Published:** 2022-09-14

**Authors:** Sunday O. Olatunji, Aisha Alansari, Heba Alkhorasani, Meelaf Alsubaii, Rasha Sakloua, Reem Alzahrani, Yasmeen Alsaleem, Mona Almutairi, Nada Alhamad, Albandari Alyami, Zainab Alshobbar, Reem Alassaf, Mehwash Farooqui, Mohammed Imran Basheer Ahmed

**Affiliations:** College of Computer Science and Information Technology, Imam Abdulrahman Bin Faisal University, P.O. Box 1982, Dammam 31441, Saudi Arabia

## Abstract

Rheumatoid arthritis (RA) is a chronic inflammatory disease caused by numerous genetic and environmental factors leading to musculoskeletal system pain. RA may damage other tissues and organs, causing complications that severely reduce patients' quality of life. According to the World Health Organization (WHO), over 1.71 billion individuals worldwide had musculoskeletal problems in 2021. Rheumatologists face challenges in the early detection of RA since its symptoms are similar to other illnesses, and there is no definitive test to diagnose the disease. Accordingly, it is preferable to profit from the power of computational intelligence techniques that can identify hidden patterns to diagnose RA early. Although multiple studies were conducted to diagnose RA early, they showed unsatisfactory performance, with the highest accuracy of 87.5% using imaging data. Yet, imaging data requires diagnostic tools that are challenging to collect and examine and are more costly. Recent studies indicated that neither a blood test nor a physical finding could early confirm the diagnosis. Therefore, this study proposes a novel ensemble technique for the preemptive prediction of RA and investigates the possibility of diagnosing the disease using clinical data before the symptoms appear. Two datasets were obtained from King Fahad University Hospital (KFUH), Dammam, Saudi Arabia, including 446 patients, with 251 positive cases of RA and 195 negative cases of RA. Two experiments were conducted where the former was developed without upsampling the dataset, and the latter was carried out using an upsampled dataset. Multiple machine learning (ML) algorithms were utilized to assemble the novel voting ensemble, including support vector machine (SVM), logistic regression (LR), and adaptive boosting (Adaboost). The results indicated that clinical laboratory tests fed to the proposed voting ensemble technique could accurately diagnose RA preemptively with an accuracy, recall, and precision of 94.03%, 96.00%, and 93.51%, respectively, with 30 clinical features when utilizing the original data and sequential forward feature selection (SFFS) technique. It is concluded that deploying the proposed model in local hospitals can contribute to introducing a method that aids medical specialists in preemptively diagnosing RA and stopping or delaying the course using clinical laboratory tests.

## 1. Introduction

Rheumatoid arthritis (RA) is a chronic inflammatory disease caused by several genetic markers, including HLA-DR4, and environmental factors, such as smoking [1]. RA is known to infect more females than males within 30 to 50 years [2], attacking the joints, especially the knees, wrists, and hands, leading to musculoskeletal system pain [3]. As smoking is the most influential environmental factor associated with RA development, other tissues and organs, such as the lungs and heart, might be affected by RA, impacting the patients' daily activities [4]. According to the Global Burden of Disease (GBD) data, the point prevalence of RA was almost 0.88 per 1000 in Saudi Arabia between 1990 and 2013 [5]. In 2021, the World Health Organization (WHO) stated that up to 1.71 billion people had musculoskeletal conditions worldwide [4]. It is recommended to identify the presence of RA within the first three months of symptoms appearing to plan for treatment procedures that reduce the illness's severity and even cure it [5]. However, RA's symptoms, including joint pain and swelling, can be challenging to detect in the early stages, as its signs are similar to those of other disorders [3]. Additionally, recent studies revealed that no disease-specific clinical features or laboratory tests could be used to diagnose it [6, 7]. Preemptive diagnosis of diseases focuses on identifying the possibility of a disease development before any symptoms appear in patients, thus, reducing or stopping the chance of developing the targeted disease in the future.

RA has traditionally been diagnosed based on the revised criteria of the 1987 American College of Rheumatology (ACR). In 2010, the ACR criteria were updated to identify patients who may develop RA based on a scale from 0 to 10. Patients are positively diagnosed with RA if their score is 6 or above [8]. However, it is observed that the 2010 criteria fail to diagnose seronegative RA [9, 10]. Besides, X-rays and magnetic resonance imaging (MRI) scans are widely utilized to identify the specific arthritis type and manage the disease progression. Although imaging facilities provide medical specialists with complete visualization of tissues involved in the development of RA, the early diagnosis of the disease remains challenging due to a lack of specificity in the findings and the limited imaging resources in some hospitals [11, 12].

Machine learning (ML) techniques can revolutionize the game by assisting doctors in diagnosing RA preemptively and accurately as they showed promising outcomes in enhancing people's quality of life and accomplishing the Kingdom's aim for health sector digital transformation [13, 14]. Few studies were conducted to diagnose RA early; most used medical imaging data; and few others used clinical data. However, the studies demonstrated unsatisfactory performance, with the highest accuracy of 87.5% using imaging data achieved by Sharon et al. [15]. Additionally, imaging data requires specialist equipment and is more challenging to manage than clinical datasets. In this study, a dataset collected from King Fahad University Hospital, Dammam, Saudi Arabia, was utilized for training three ML algorithms, namely, support vector machine (SVM), logistic regression (LR), and adaptive boosting (Adaboost). The models were then combined in a voting ensemble to get the maximum predictive performance [16]. The base classifiers were chosen carefully for the following reasons: SVM is known for its promising results in predicting various chronic diseases [17]; LR is simpler to implement, analyze, and train; and Adaboost is known for increasing diagnostic accuracy [18].

This study conducted two experiments utilizing the three aforementioned ML algorithms to build the novel voting ensemble. In the first experiment, the algorithms were trained using the original data. The second experiment applied the synthetic minority oversampling technique (SMOTE) to the training dataset to balance the classes. A voting ensemble was built in each experiment using multiple versions of the trained traditional classifiers. Afterward, two feature selection techniques were utilized to discover the ideal feature subsets that deliver the most outstanding performance for each algorithm, including sequential forward feature selection (SFFS) and sequential backward feature selection (SBFS). The empirical results indicated that voting model outperformed all other classifiers, achieving the highest accuracy of 94.03% when utilizing the original data and SFFS technique. Furthermore, it is proved that the proposed voting ensemble demonstrated promising outcomes in the preemptive diagnosis of RA, with a recall and precision of 96.00% and 93.51%, respectively, using 30 features. It is also revealed that the combination of the laboratory tests utilized in this study could aid medical specialists in the early diagnosis of RA.

In this paper, the remaining parts are organized into sections. The literature review is discussed in Section 2, whereas Section 3 compromised the materials and methods used. Moreover, Section 4 evaluated the experiment outcomes. Lastly, Section 5 presented the conclusion and future work recommendations.

### 1.1. Contribution

This study aims to develop a robust tool for the preemptive diagnosis of RA that could be utilized by local hospitals, even with limited capabilities. The contributions of this study are as follows:

- Implement a novel voting ensemble that achieves a high classification accuracy for the preemptive diagnosis of RA to assist medical specialists before any symptoms appear
- Reduce the possible complications of the late-stage identification of RA
- Investigate the possibility of diagnosing RA preemptively using clinical laboratory tests
- The proposed model generally achieved the highest outcomes compared to the benchmark studies

## 2. Review of Related Literature

RA is one of the most dangerous chronic diseases leading to progressive joint damage. The early treatment of RA plays an essential role in inhibiting severe symptoms that can affect the patients' quality of life. Therefore, it is crucial to aid rheumatologists in detecting RA early to prevent its progression. As shown below, intensive work has been carried out by utilizing supervised and unsupervised ML techniques to detect the presence of RA in patients using clinical and imaging data.

Morita et al. [19] developed a computer-aided diagnosis system using ML algorithms to predict RA with image data. The dataset contained 45 hand X-ray images (mild-to-severe) of RA patients. After applying some image processing techniques, the dataset records increased to 6,300 image patches for each class (positive and negative). SVM and support vector regression (SVR) were used to detect finger joint and estimate the mTS score, respectively. The outcomes exhibited that SVM achieved an accuracy of 81.4%, whereas SVR attained 50.9% for estimating erosion and 64.3% for joint space narrowing (JSN) scores.

In another study, Sharon et al. [15] utilized Weka to apply ML techniques for the early prediction of RA. The authors used a thermal imaging dataset containing eight attributes and 32 instances. SVM and random forest (RF) were used as weak classifiers to train three ensemble classifiers: Adaboost, bagging, and subspace. The results revealed that Adaboost combined with RF achieved the best results with an accuracy of 87.5%, precision of 87.3%, recall of 87.5%, and ROC of 0.718.

Likewise, Sharon et al. [20] explored ensemble techniques for classifying RA images using two datasets. The first dataset included 40 records and 9 attributes, whereas the second consisted of 310 instances and 6 features. The empirical results showed that using the first dataset, random subspace combined with *K*-nearest neighbors (K-NN) attained the highest accuracy of 97.50% with 10-fold cross-validation and 66.67% using the holdout evaluation technique. On the other hand, the results revealed that using the second dataset, bagging with RF achieved the highest accuracy of 94.84% with 10-fold cross-validation and 83.81% using the holdout validation technique. Despite the high accuracy attained using the training set, the proposed models showed unsatisfactory results using the unseen data.

On the other hand, Yoo et al. [21] focused on predicting RA using the *K*-means clustering technique. A clinical dataset including 60 anonymous patient records was obtained from the Eulji University Hospital. The *K*-means clustering was used to predict the rheumatoid factor, anticyclic citrullinated peptides, swollen joint count (SJC), and erythrocyte sedimentation rate (ESR) thresholds to forecast whether a patient has developed RA. The empirical results demonstrated that the *K*-means clustering achieved an accuracy of 84%. Moreover, the results indicated that RA could be classified as two or four factors.

Similarly, Singh et al. [22] used the same dataset with three clustering techniques to detect RA, including *K*-means, hierarchical, and density-based spacial clustering of applications with noise (DBSCAN). Moreover, the authors compared the techniques' execution time, in which the results showed that DBSCAN and *K*-means had similar time complexity O(*n*^2^), whereas the hierarchical algorithm had O(*n*^3^).

Furthermore, Shanmugam and Preethi [23] proposed a framework for predicting RA using clinical and genetic factors by employing ML and data mining techniques. The authors utilized a dataset with 9 features obtained from the Coimbatore Government Medical College. They selected 5 of 9 attributes ranked by physicians. Later, they individually implemented Naive Bayes (NB), SVM, artificial neural network (ANN), and Adaboost algorithms and combined them via an ensemble voting algorithm. The results showed that Adaboost attained the highest accuracy of 85%.

The reviewed studies showed unsatisfactory performance of the proposed models in the early diagnosis of RA. The highest outcome was achieved by Sharon et al. [15] with an accuracy of 87.5% using imaging data. Medical imaging data requires specialized equipment to be collected and is more complex to handle than tabular datasets. In addition, as far as we know, no studies have been conducted on the preemptive prediction of RA. Accordingly, this study aims to utilize clinical and demographical data as they are less expensive and easier to access and examine than imaging data, hence, reducing the demand for acquiring expensive imaging technologies and enabling local hospitals with no imaging facilities to diagnose RA preemptively.

## 3. Materials and Methods

This study built RA diagnosis models using the Python programming language with a constant random_state value of 42 for all operations. Two datasets obtained from King Fahad University Hospital (KFUH) were merged, and various preprocessing techniques were applied to them. The merged dataset was then divided into a stratified ratio of 70% for training and validation and 30% for testing. After splitting the dataset, the min-max scaler was fitted to the training set and transformed to the testing set. Subsequently, two experiments were conducted using three ML algorithms, namely, support vector machine (SVM), logistic regression (LR), and adaptive boosting (Adaboost), trained with all features. In the first experiment, the algorithms were trained using the original data. In the second experiment, the synthetic minority oversampling technique (SMOTE) was applied to the training set to balance the classes. GridSearchCV was then utilized to optimize the hyperparameters of SVM, LR, and Adaboost using stratified 10-fold cross-validation for both experiments. Successively, a voting ensemble model was constructed in each experiment using different versions of the trained traditional classifiers. The forward and backward sequential feature selection techniques were then applied to the classifiers and voting ensemble to achieve the best performance while lessening the number of features. The final models were evaluated in terms of several performance measures, including accuracy, precision, recall, and receiver operating characteristic (ROC).  Figure 1 summarizes the steps followed to build the prediction models.

### 3.1. Description of Dataset

The dataset utilized to perform this experiment was driven by integrating two clinical RA datasets obtained from King Fahad University Hospital (KFUH), Dammam, Saudi Arabia. The first dataset contained 196 instances and 45 features, while the second comprised 262 samples and 39 attributes. The columns were selected considering the ratio of missing values within each column, not exceeding 30%. Additionally, few instances were excluded due to the overabundance of the missing data. As a result of incorporating equivalent features from both datasets, the resultant dataset comprised 31 attributes and 446 instances, including 251 positive cases of RA and 195 negative cases of RA.  Table 1 describes the features used in this study.

This study aimed to investigate whether it is possible to diagnose RA preemptively using clinical laboratory markers used to track RA progression and other clinical tests. A commonly used blood test for the diagnosis of RA is the complete blood count (CBC), measuring WBC, RBC, HCT, HGB, and platelet counts. Similarly, the complete metabolic panel (CMP) estimates the level of SGOT, GGTP, sodium, potassium, chloride, glucose, and creatinine in the blood to assess liver and kidney functions [24, 25]. Both CBC and CMP are utilized as indicators for the general health of the patients and the disease activity, making their results indispensable in the prediction of RA.

### 3.2. Statistical Analysis

The statistical analysis tools assist in identifying the essential information that aids in performing the proper preprocessing techniques before beginning modeling. The statistical analysis for the numerical attributes present in the dataset is shown in Table 2, including the count, mean, standard deviation, and the five-number summary for each feature. Besides, Figure 2 illustrates the correlation between the variables and the target class. It is concluded that the age and sex attributes are the most correlated features with the target class since RA is more prevalent in females and the age ranges between 30 and 50 [2, 26]. Moreover, it is revealed that the platelet count and MPV features are more correlated with the target class than the other clinical tests in the dataset.

### 3.3. Preprocessing

Data preprocessing is one of the essential steps carried out in order to make raw data usable and efficient. In the present study, several preprocessing techniques were conducted using Python's Sklearn and Pandas libraries. Numeric inputs and outputs are compulsory for machine learning models. Hence, categorical data must be encoded into numbers before training and evaluating a model. In this experiment, we converted the categorical variables to numeric by setting the majority label to 1 and the other to 0, as represented in

(1) $$\begin{array}{c} x_{i}=\text{mode}\left\{x_{1},x_{2},\cdots ,\cdots ,x_{n}\right\},x_{i}=1, \end{array}$$

(2) $$\begin{array}{c} x_{i}\neq \text{mode}\left\{x_{1},x_{2},\cdots ,\cdots ,x_{n}\right\},x_{i}=0, \end{array}$$

where *x*_*i*_  is the *i*^*th*^ value in a categorical feature.

Machine learning algorithms are highly affected by the distribution of the dataset. Outliers are one of the issues that could negatively affect the statistical power by introducing skewness and bias that negatively impact a model's performance. In this study, the outliers were calculated using the interquartile range (IQR) technique. Any value above or below bounds is substituted with the median value, as shown in

(3) $$\begin{array}{c} \text{Lower bound}=Q1-3\times \left(Q3-Q1\right), \end{array}$$

(4) $$\begin{array}{c} \text{Upper bound}=Q3+3\times \left(Q3-Q1\right), \end{array}$$

(5) $$\begin{array}{c} \text{Lower bound}>x_{i}>\text{Upper bound},x_{i}=\frac{n+1}{2}\text{term}, \end{array}$$

where *Q*1 represents the first quartile, *Q*3 denotes the third quartile, *x*_*i*_  is the *i*^*th*^ value in a feature, and *n* is the number of values in a column.

Data skewness is caused by an uneven distribution of data, causing a curve to appear deformed to the left or right. An ML model is less capable of describing typical cases since it must cope with rare cases on extreme values. Accordingly, the columns with skewness greater than 0.5 are treated in this study using the cubic transformation technique, represented in the following equation, where *f*_*i*_ is the *i*^*th*^ feature in the dataset.

(6) $$\begin{array}{c} f_{i}=\sqrt[{3}]{f_{i}}. \end{array}$$

Missing values impose a significant effect on the conclusions driven from the dataset. Some of the various problems missing values cause are statistical power reduction, biased parameters estimation, and data analysis complications. Imputation approaches to these values differ based on the attribute types. In this study, the missing numerical values were imputed using the mean value, as shown in the following equation , where *X* represents a data point and *n* denotes the total number of values in a column.

(7) $$\begin{array}{c} \text{Mean}=\frac{\sum X}{n}. \end{array}$$

After applying the preprocessing techniques, the dataset was divided into a stratified ratio of 70 : 30, where 70% of the data was used for training and validation, and the remaining was used for testing. After splitting the dataset, the min-max scaler was fitted to the training set and transformed to the testing set to scale the data between 0 and 1 using

(8) $$\begin{array}{c} \text{MinMaxScaler }\left(v^{\prime }i\right)=\frac{x_{i}-\min_{A}}{\max_{A}-\min_{A}}\left(\text{ne}{\text{w}}_{\max_{A}}-\text{ne}{\text{w}}_{\min_{A}}\right)+\text{ne}{\text{w}}_{\min_{A}}, \end{array}$$

where *x*_*i*_ denotes the *i*^*th*^  value, max_*A*_ and min_*A*_ represents a feature's maximum and minimum values, and *new*_max_*A*_ and *new*_min_*A*_ are the values 0 and 1, respectively.

### 3.4. Description of the Proposed Techniques

This section describes the utilized ML algorithms, including SVM, LR, and Adaboost.

#### 3.4.1. Support Vector Machine (SVM)

Support vector machine (SVM) is a robust supervised ML algorithm employed in classification and regression tasks with its primary use in classification. SVM became popular after the introduction of its concept by Cortes and Vapnik in the late 1990s [27]. It is known for its capability to handle both linear and nonlinear data. For linearly separable data, SVM classifies the data points by finding an optimal decision boundary, known as the hyperplane, with the maximum margin distance in an *N*-dimensional space. The hyperplane is constructed using Equation (9), whereas the points are placed to the left or right of the hyperplane using the following equations [28]:

(9) $$\begin{array}{c} w^{T}x_{i}+b=0, \end{array}$$

(10) $$\begin{array}{c} w^{T}x_{i}+b>0,y_{i}=1, \end{array}$$

(11) $$\begin{array}{c} w^{T}x_{i}+b<0,y_{i}=-1, \end{array}$$

where *w* denotes the weight vector, *x* the input vector, and *b* the bias.

Finding the optimal hyperplane for a better classification requires a maximization of the margin. It can be granted by minimizing the weight vector. Thus, obtaining generalization control, Equation (12) shows the constrained optimization problem for computing the maximum marginal hyperplane (MMH) [29].

(12) $$\begin{array}{c} \mathrm{minimize}=\frac{1}{2}{\left\|w\right\|}^{2}, \end{array}$$

(13) $$\begin{array}{c} \text{subject to }y_{i}\left(\left\langle w∙\left.x\right\rangle \right.+b\right)>0. \end{array}$$

SVM employs a kernel function to solve nonlinear data by adding more dimensions to the data to make it linear in a higher-dimensional space [30].

#### 3.4.2. Logistic Regression (LR)

Logistic regression (LR) is a popular statistical-based supervised ML algorithm commonly used for classification problems. David Cox developed it in 1958 and named it LR because it uses a logistic function as the processes' core. LR is famous for its simplicity and efficiency in solving linear and binary classification problems while achieving outstanding performance for linearly separable data [31]. It utilizes a sigmoid function, also referred to as a logistic function, which has an S-shaped curve to transform the data values to the range [0,1] [32]. The following equation represents the formula for calculating the sigmoid function [33].

(14) $$\begin{array}{c} \text{Sigmoid function }\left(t\right)=\frac{1}{1-e^{-x}}, \end{array}$$

where *x* is a linear function calculated using [33]

(15) $$\begin{array}{c} x=\left(b_{0}+b_{1}x\right). \end{array}$$

LR produces probabilistic values between 0 and 1 to predict a categorical dependent attribute using several independent attributes by employing the concept of setting a threshold value. The threshold is responsible for mapping the prediction probability to either 0 or 1 [31]. Afterward, if the outcome is greater than or equal to the threshold, it will be labeled as a positive class. Otherwise, it will be considered a negative class.

#### 3.4.3. Adaptive Boosting (Adaboost)

Adaptive boosting (Adaboost) is a dependent ensemble method applied in classification tasks. It is one of the best statistical classifiers introduced in 1997 by Freund and Schapire [34]. Adaboost is a fast, compatible, and simple technique that can achieve high accuracy and avoid overfitting by providing good generalization control [35]. The primary use of Adaboost is to improve the performance of the decision tree algorithm in binary classification cases [36]. Accordingly, Adaboost utilizes multiple weak learners in several iterations to correctly categorize the misclassified samples from the previous weak classifier. For each learner, the misclassified data points' weights are boosted, while correct samples' weights are decreased per iteration through the training. Consequently, the results of each model are combined to form one strong learner with the best performance and slightest error [37]. The following equation represents Adaboost's classification approach, where *h* represents the weak classifier and *α* denotes its corresponding weight [38].

(16) $$\begin{array}{c} H\left(X\right)=\mathrm{sign}\;\left(\overset{T}{\underset{t=1}{\sum }}\alpha_{t}h_{t}\left(x\right)\right). \end{array}$$

### 3.5. Performance Measures

This study utilized three performance measures to evaluate and compare the built models' performance: accuracy, precision, and recall. Accuracy is the most popular measure, which measures the rate of accurate predictions formed by the models. On the other hand, precision calculates the number of actual positive predicated instances classified correctly to positive samples, and recall calculates the number of positive cases classified correctly.

(17) $$\begin{array}{c} \text{Precision}=\frac{\text{Correctly classified as RA}}{\text{Correctly classified as RA}+\text{Incorrectly classified as RA}},\\ \text{Recall}=\frac{\text{Correctly classified as RA}}{\text{Correcly classified as RA}+\text{Incorrectly classified as Non}-\text{RA}},\\ \text{Accuracy}=\frac{\text{Correctly classified as RA}+\text{Correctly classified as Non}-\text{RA}}{\text{Total prediction results}}. \end{array}$$

Additionally, ROC curves were constructed to measure the models' performance in distinguishing between different classes. It calculates each model's accuracy by comparing the actual positive rate versus the false-positive rate with various thresholds [10].

### 3.6. Optimization Strategy

GridSearchCV used a grid of parameters to perform hyperparameter tuning by testing the effectiveness of classifiers that were constructed using various combinations of hyperparameters. GridSearchCV aims to find the optimal combination of hyper-parameters values that generate the best results for each classifier, leading to enhanced results [39, 40].

In both experiments, the SVM hyper-parameters grid comprised cost, Gamma, and kernel. The cost included the values {1, 2, 3, 4, 5, 6, 7, 8, 9, 10, 15, 20, 25, 30}, whereas the Gamma included the values {1, 0.1, 0.01, 0.001, 0.0001, scale, auto}. Moreover, the grid contained the kernel functions {RBF, Sigmoid, Linear, Polynomial}.

Furthermore, the hyperparameter grid for LR included cost, penalty, and solver. The cost values compromised {1, 2, 3, 4, 5, 6, 7, 8, 9, 10, 15, 20, 25}, while the penalty consisted of the values {none, L1, L2}. Moreover, the grid contained the solver values {Newton-cg, Lbfgs, Liblinear, Sag, Saga}.

Additionally, the hyperparameter grid for Adaboost contained N_estimators and Learning_rate. The N_estimators values included {10, 20, 30, 40, 50, 60, 70, 80, 90, 100, 150, 200, 250}, while the Learning_rate consisted of the values {0.0001, 0.001, 0.01, 0.1}. The sections below represent the results of applying GridSearchCV on the original and upsampled data.

#### 3.6.1. Optimizing the Algorithms Using the Original Data

Each graph in Figure 3 illustrates the performances of the SVM classifier using different kernel functions with distinct cost and Gamma values. It is indicated that there was a competitive performance between Gamma values 0.1 and auto using the RBF and sigmoid kernels. It was also revealed that the Gamma value 0.1 provided the best performance for SVM using the polynomial (Poly) kernel. Moreover, it can be observed that the change in the Gamma value did not influence the linear kernel as the values are overlapping. Overall, in combination with Gamma value one and cost value five, the linear kernel yielded the highest validation accuracy of 85.90%.

The performances of LR using different penalty values along with various cost and solver values are presented visually in Figure 4. It is indicated that the saga solver enhanced LR outcomes when combined with all penalties. Apart from that, it is revealed that the Newton-cg and Liblenear solvers improved LR's results when combined with the none penalty and L2 penalty, respectively. The L1 penalty combined with a cost value of 1 and the saga solver generated the validation highest accuracy of 85.90%.

Figure 5 displays the performance of Adaboost using different N_estimators and Learning_rate values. Overall, it is indicated that the Learning_rate value of 0.1 improved the performance of Adaboost significantly compared to the other Learning_rate values. However, when the N_estimator's value increased to 200, the other Learning_rate values outperformed the value 0.1. Moreover, it is revealed that the Learning_rate values 0.001 and 0.0001 did not affect Adaboost's outcomes. The highest validation accuracy of 84.61% was achieved when the Learning_rate and N_estimators values were 0.1 and 80, respectively.

#### 3.6.2. Optimizing the Algorithms Using the Upsampled Data

Each graph in Figure 6 exhibits the performances of the SVM classifier using several kernel functions with different cost and Gamma values after upsampling the data. It is indicated that there was a competitive performance between Gamma values 0.1 and auto using the RBF kernel. On the other hand, the auto Gamma outperformed when combined with the sigmoid kernel, whereas the 0.1 Gamma surpassed when combined with the poly kernel. Moreover, it can be observed that the change in the Gamma value did not influence the linear kernel as the values are overlapping. Overall, in combination with Gamma value 0.1 and cost value 5, the RBF kernel yielded the highest validation accuracy of 87.49%.

The performances of LR using different penalty values along with various cost and solver values after upsampling the dataset are presented visually in Figure 7. It is indicated that the saga solver enhanced LR outcomes when combined with all penalties. Additionally, it is revealed that the Newton-cg and Lbfgs solvers improved LR's results when combined with the L2 penalty. The L2 penalty combined with a cost value of 3 and the Newton-cg solver generated the highest validation accuracy of 87.77%.

Figure 8 displays the performance of Adaboost using different N_estimators and Learning_rate values. It is observed that the 0.1 Learning_rate enhanced Adaboost's performance considerably compared to other Learning_rate values. Additionally, it is revealed that the Learning_rate values 0.001 and 0.0001 did not affect Adaboost's outcomes. The highest validation accuracy of 86.06% was achieved when the Learning_rate and N_estimators values were 0.1 and 100, respectively.

Table 3 summarizes the proposed classifiers' performance with their optimal hyperparameters and validation accuracy. It is concluded that the SMOTE improved the performance of the techniques in terms of validation accuracy.

### 3.7. Proposed Voting Ensemble

Ensemble approaches exploit the strengths of weak learning algorithms to create a robust and efficient model. They have a superior ability to deal with complex problems than single classifiers, as ensemble models can solve the diversities produced by the single algorithms more efficiently [41]. A voting classifier is an ensemble ML algorithm utilized for classification tasks. It combines the outcomes of different ML classifiers to achieve a better predictive performance than an individual classifier. Moreover, it produces the class prediction based on the classifiers' majority of voting [42]. There are two popular voting types in a voting classifier: hard voting and soft voting. In hard voting, the final prediction is the class that acquires the most voting from the classifiers. In contrast, in soft voting, the predicted class is the class that achieves the highest average of probability assigned to it by the classifiers [43]. In this study, the hard voting approach is used, as shown in Equation (18), where ${\hat{y}}_{f}$ is the final prediction, *C*_*i*_ are the predictions of *i*^th^ observations, and *x* is the data sample [44].

(18) $$\begin{array}{c} {\hat{y}}_{f}=\text{mode }\left\{C_{1}\left(x\right),C_{2}\left(x\right),\cdots ,C_{n}\left(x\right)\right\}. \end{array}$$

The creation of the proposed novel model was implemented in two experiments without and with applying SMOTE to the dataset. Since the GridSearchCV results varied in the two experiments, the implementation of the voting models differed in both experiments. However, in both proposed models, 7 classifiers were employed. The first experiment's novel voting ensemble incorporated the best three SVM models obtained by the GridSearchCV since SVM attained the highest testing accuracy. Additionally, it contained two versions of LR and Adaboost models as they achieved similar testing accuracies. On the other hand, the second experiment's proposed model comprised the best three versions of SVM and LR models produced by the GridSearchCV along with one Adaboost model due to its low performance on the testing data, which might degrade the performance of the voting ensemble.  Figure 9 shows the constructed novel models' summary along with their hyperparameters.

## 4. Results and Discussion

This study conducted two experiments to train three ML algorithms and propose the novel voting ensemble model using a stratified 70 : 30 percentage. In the first experiment, the algorithms and voting ensemble were trained using the original dataset that suffers from the class imbalance issue. On the other hand, the second experiment utilized the SMOTE technique to balance the dataset, in which the algorithms and proposed voting ensemble were trained using the upsampled dataset.  Table 4 compares each experiment's model performance with its optimal hyperparameters obtained from the GridSearchCV method.

As shown in Table 4, the proposed voting ensemble outperforms the traditional classifiers in experiment 1, attaining a classification accuracy of 94.03%, followed by SVM, achieving 93.28%. In terms of precision, the proposed voting ensemble achieved the highest score of 93.51%, followed by SVM and Adaboost, scoring 93.42% and 93.24%, respectively. Additionally, the proposed voting technique surpassed the traditional algorithms outstandingly, scoring 96.00% in terms of recall. LR attained the most undesirable outcome in terms of accuracy and precision, scoring 91.04% and 89.87%, respectively. However, it achieved a remarkable recall score of 94.67%.

Opposingly, in experiment 2, the proposed voting ensemble and LR outperformed other models in terms of accuracy and recall, achieving 93.28% and 94.67%, respectively. Adaboost attained the highest precision among the other classifiers, scoring 94.20%. However, it demonstrated a weak performance in terms of accuracy and recall, scoring 89.55 and 86.67%, respectively.

Generally, the results verified competitive performance using the original and upsampled data. It is indicated that SVM, LR, and the proposed voting model performed better using the original data in terms of recall and accuracy, with a notable difference compared to the performance using the upsampled data. Conversely, it is revealed that SMOTE enhanced the LR results in terms of all the performance measures, except the recall, in which it yielded the same score. To further assess the credibility of the attained results, the irrelevant variables will be eliminated from each algorithm using two feature selection techniques, as presented in the upcoming section.

### 4.1. Feature Selection

Feature selection is considered to have a vital role in building an excellent prediction classifier. It produces a superior prediction accuracy using the minimum set of features that decreases the computational complexity. In this study, two feature selection techniques, namely, sequential forward feature selection (SFFS) and sequential backward feature selection (SBFS), were utilized to find an optimal feature subset that yields the best performance for each classifier. The SFFS technique begins from an empty set of features, and an attribute is added to the set at each step if it maximizes the classifier's accurate predictions [45]. In contrast, the SBFS technique uses all of the features to build the classifier in the first step and then builds several classifiers iteratively, eliminating one attribute at a time until an optimal feature subset is obtained [45]. Tables 5 and 6 demonstrate the performance of the classifiers after applying the sequential forward and backward feature selection techniques.

It is revealed from Table 5 that the SFFS technique in experiment 1 reduced SVM's and Adaboost's classification accuracy by 3.73% and 2.98%, respectively. However, it maintained the same performance of LR and voting with fewer features. On the other hand, it is denoted that the SFFS technique degenerated the accuracy of SVM, Adaboost, and voting in experiment 2 by 2.98%, 3.73%, and 2.24%, respectively, while preserving the same performance of LR using less number of features.

It is observed from Table 6 that the SBFS technique slightly degenerated the accuracy of SVM, Adaboost, and voting in experiment 1 by 0.74%, 0.75, and 0.75%, respectively. Conversely, it maintained the accuracy of LR while somewhat lessening the number of features to 31. On the other hand, it is noted that the SBFS technique decreased the classification accuracy of LR and voting in experiment 2 by 0.74%. Opposingly, it improved the performance of Adaboost by increasing the accuracy by 2.99% with six attributes while maintaining the performance of SVM with 22 attributes.

Comparing the performance of models trained using the original and upsampled data with the sequential forward and backward feature selection techniques, it is concluded that the proposed voting ensemble attained the highest accuracy when utilizing the original data and SFFS technique. Besides, LR performed best using the upsampled data and SFFS technique. On the contrary, Adaboost achieved the best performance using the upsampled data with the SBFS technique. Although SVM's accuracy was reduced when applying feature selection techniques in both experiments, it is suggested that SVM performed better using the original data and SFFS technique. The reason behind the conclusion is that it achieved the same recall value, as shown in Table 7, with a slight reduction in accuracy and fewer features.

### 4.2. Further Discussions

Chronic diseases are the primary cause of disability, morbidity, and fatalities, threatening humans' lives and the country's economy [46]. RA is an example of a chronic inflammatory disease that attacks patients' joints and causes musculoskeletal system pain. The late diagnosis of the disease causes structural damage, which is highly associated with more significant functional disability [47]. Nowadays, ML applications are widely used for early diagnosis and progression management of chronic diseases to empower specialists in making better and faster decisions [48]. Moreover, it is evident that ML is taking on increasing relevance in clinical laboratory medicine due to the widespread accessibility of open-source tools and the decreased cost of collecting and storing data using laboratory automation [49]. Hence, developing a diagnosis system for the preemptive prediction of RA using state-of-art AI technologies is worth researching. This study constructed a novel voting ensemble using SVM, LR, and Adaboost with clinical laboratory tests. Table 7 compares the best versions of the proposed voting ensemble and traditional algorithms.

Table 7 indicates that the proposed voting model achieved outstanding performance in terms of recall, scoring the highest value of 96.00%. On the other hand, Adaboost outperformed the proposed model in terms of precision, scoring 95.77%. A high precision score ensures fewer false-positive cases. Reducing false-positive cases can avoid anxiety, unnecessary diagnostic and therapeutic procedures, and increased costs and risks [50]. On the other hand, a high recall score guarantees fewer false-negative tests. The increment in false-negative cases may lead to severe consequences, leading to the rapid advancement of disease progression that may lower the patients' chances of recovery. In addition, it could lead to serious legal action resulting in costly payments. Hence, it is more crucial to ensure the minimum presence of false negative to reduce the impact of such consequences [51]. A confusion matrix is considered a reliable metric for determining how accurate the classification algorithm is, in which a good model will always have high precision and recall [52]. Therefore, for further analysis of false-positive and false-negative cases, confusion matrices are constructed for the best-performing models and displayed in Figure 10, which are the versions of SVM and voting without sampling, and the versions of LR and Adaboost trained using the upsampled data.

It is crucial to consider the values given by the confusion matrix, primarily focusing on false negative to avoid severe consequences. It is indicated that the proposed voting achieved the lowest false negative of 3, whereas Adaboost yielded the highest false-negative value of 7. Voting produced the exact false-positive count as LR. Yet, the proposed voting ensemble is preferred due to the higher value of true positive, showing the model's correct classification of RA patients with the fewest false-negative cases.

Further analysis is done using the area under receiver operating characteristics (AUROC), as illustrated in Figure 11, to prove the ability of the proposed model to discriminate between the classes. The ROC curves were generated using stratified 10-fold cross-validations to evaluate the performance of LR and Adaboost after sampling and SVM and voting before sampling.

It is revealed that the highest AUC value of 0.94 was achieved by voting, followed by an approximate AUC value of 0.93 obtained from both LR and Adaboost models, whereas SVM attained the lowest AUC value of 0.92. This analysis clarifies that voting scored the best AUC value, proving its reliability in diagnosing RA patients accurately with fewer errors than the traditional algorithms. In comparison to the benchmark studies, most of the studies utilized imaging datasets for the early prediction of RA, scoring below 90%, which is impractical in medical applications. Sharon et al. [15] proposed an ensemble model trained using two imaging datasets, which attained an accuracy of 97.50% and 94.84% using 10-fold cross-validation. However, the model was not generalizable while using the holdout validation technique, achieving 66.67% and 83.81%. To the best of our knowledge, only one study experimented with clinical and genetic factors, attaining accuracy of 85% [23]. The proposed ensemble model in this study outperformed the benchmark models achieving an accuracy, recall, and precision of 94.03%, 96.00%, and 93.51%, respectively, with 30 clinical features.

## 5. Conclusion and Recommendation

A delayed diagnosis of RA can lead to progressive damage to joints, tissues, and organs. In this study, two experiments were carried out to achieve outstanding performance in diagnosing RA preemptively. For the first experiment, algorithms were trained using original data, while for the second experiment, SMOTE was used to balance the training dataset. In both experiments, three ML algorithms, including SVM, LR, and Adaboost, were trained using a Saudi clinical dataset obtained from King Fahad University Hospital to diagnose rheumatoid arthritis (RA) preemptively. A novel ensemble was then assembled using different versions of the traditional classifiers. Subsequently, two feature selection strategies, sequential forward feature selection and sequential backward feature selection, were used to determine an optimal feature subset that provides the best performance for each algorithm. The study findings indicated that the proposed voting ensemble provides promising diagnosis outcomes. It outperformed other traditional classifiers with accuracy, recall, and precision of 94.03%, 96.00%, and 93.51%, respectively, with 30 features when utilizing the original data and sequential forward feature selection technique. Hence, it is presumed that our findings can improve people's quality of life and delay or stop the disease's course before the symptoms appear within the early months.

This paper encourages the further expansion of the work by including more RA datasets from other repositories to explore clinical laboratory tests that are more correlated with the target class. Additionally, other feature selection techniques could be investigated to reduce the number of features required to attain reliable outcomes. The possibility of enhancing the results could also be attempted by extending the proposed voting ensemble to incorporate more classifiers.

## Figures and Tables

**Figure 1:** Rheumatoid arthritis prediction framework.

**Figure 2:** Correlation heatmap.

**Figure 3:** (a) RBF kernel; (b) sigmoid kernel; (c) linear kernel; and (d) poly kernel.

**Figure 4:** (a) None penalty; (b) L1 penalty; and (c) L2 penalty.

**Figure 5:** Adaboost hyperparameter tuning.

**Figure 6:** (a) RBF kernel; (b) sigmoid kernel; (c) linear kernel; and (d) poly kernel.

**Figure 7:** (a) None penalty; (b) L1 penalty; and (c) L2 penalty.

**Figure 8:** Adaboost hyperparameter tuning.

**Figure 9:** Proposed voting ensemble (a) experiment 1 and (b) experiment 2.

**Figure 10:** (a) SVM confusion matrix; (b) LR confusion matrix; (c) Adaboost confusion matrix; and (d) voting confusion matrix.

**Figure 11:** (a) SVM AUROC; (b) LR AUROC; (c) Adaboost AUROC; and (d) voting AUROC.

**Table 1:** Dataset description.

Feature	Description
Sex	Male or female.
Age	Age of the patient in years.
Mean corpuscular hemoglobin (MCH)	The hemoglobin's average amount in a red blood cell.
Mean corpuscular volume (MCV)	The average size of red blood cells.
Mean corpuscular hemoglobin concentration (MCHC)	The hemoglobin concentration in a given volume of a red blood cell.
Red cell distribution width (RDW)	The variance in size and volume of red blood cells.
Platelet count	The number of platelets in the body.
Mean platelet volume (MPV)	The average size of platelets.
Hemoglobin (HGB)	The amount of HGB in red blood cells.
Hematocrit (HCT)	The red blood cells proportion in the blood.
White blood cells (WBC)	The WBC count in the blood.
Red blood cells (RBC)	The RBC count in the blood.
Monocytes (MONO)%	The percentage of a particular type of WBCs.
Monocytes (MONO)#	The absolute count of a particular type of WBCs.
Eosinophils (EOS)%	The percentage of eosinophils in WBCs.
Eosinophils (EOS)#	The absolute count of eosinophils in WBCs.
Neutrophil (NEU)%	The percentage of neutrophils in WBCs.
Neutrophil (NEU)#	The absolute count of neutrophils in WBCs.
Lymphocytes (LYMPH)%	The percentage of lymphocytes in the blood.
Lymphocytes (LYMPH)#	The absolute count of lymphocytes in the blood.
Basophils (BASO)%	The percentage of basophils in the blood.
Basophils (BASO)#	The absolute count of basophils in the blood.
SODIUM	The amount of sodium in the blood.
Potassium	The amount of potassium in the blood.
Chloride	The amount of chloride in the blood.
Carbon dioxide (CO2)	The amount of CO2 in the blood.
Anion gap	The measurement of acid-base balance in the blood.
Gamma-glutamyl transferase (GGTP)	The amount of GGTP in the blood.
Alkaline phosphatase (ALP)	The measurement of ALP in the blood.
Serum glutamic-oxaloacetic transaminase (SGOT)	The measurement of aspartate aminotransferase (AST) enzyme in the blood serum.
Serum glutamic pyruvic transaminase (SGPT)	The amount of glutamate pyruvate transaminase (GPT) in blood serum.

**Table 2:** Statistical analysis of numerical features.

Feature	Mean	Standard deviation	Minimum	25%	50%	75%	Maximum	Missing values
Age	57.54	14.86	17.00	48.00	58.00	68.00	92.00	1.00
MCH	26.79	3.36	14.00	25.00	27.05	29.00	36.20	13.00
MCV	81.55	8.09	48.00	77.15	82.70	87.00	106.50	14.00
MCHC	32.77	1.43	25.00	32.00	33.00	33.90	36.00	14.00
RDW	15.19	2.39	12.00	13.70	14.50	16.00	26.70	14.00
Platelet count	278.09	92.43	53.00	213.00	268.00	329.00	664.00	14.00
MPV	9.34	1.20	6.00	8.40	9.30	10.20	13.10	22.00
HGB	12.30	1.91	7.00	11.20	12.40	13.58	17.30	15.00
HCT	37.55	5.25	20.30	34.70	37.80	41.10	50.80	15.00
WBC	7.45	3.45	0.73	5.30	6.60	8.90	28.35	35.00
RBC	4.62	0.70	2.14	4.18	4.65	5.06	7.24	33.00
MONO%	8.68	2.46	1.00	7.00	8.60	10.20	18.50	24.00
EOS%	3.30	2.56	0.00	1.70	2.70	4.20	18.00	24.00
NEU%	53.09	13.61	14.00	43.98	52.85	61.90	93.00	25.00
LYMPH%	34.12	12.38	1.00	26.15	33.55	42.13	78.00	25.00
BASO%	0.60	0.36	0.00	0.30	0.50	0.80	2.20	25.00
BASO#	0.03	0.05	0.00	0.00	0.00	0.10	0.40	28.00
SODIUM	139.07	3.13	117.0	137.00	139.00	141.00	146.00	23.00
NEU#	4.00	2.22	0.70	2.40	3.50	5.10	13.60	26.00
LYMPH#	2.34	1.18	0.20	1.70	2.20	2.80	18.50	28.00
MONO#	0.61	0.25	0.10	0.40	0.60	0.70	2.20	28.00
EOS#	0.23	0.23	0.00	0.10	0.20	0.30	2.20	29.00
Potassium	4.29	0.48	2.90	4.00	4.30	4.60	6.40	27.00
Chloride	102.81	3.00	82.00	101.00	103.00	105.00	111.00	27.00
CO2	27.40	3.12	6.00	26.00	28.00	29.00	38.00	70.00
Anion gap	8.64	2.79	1.00	7.00	9.00	10.00	29.00	61.00
GGTP	51.92	69.29	11.00	23.00	33.50	48.25	838.00	81.00
ALP	85.07	54.89	11.00	61.00	74.00	95.00	703.00	46.00
SGOT	26.51	32.10	7.00	16.00	21.00	27.00	442.00	48.00
SGPT	31.52	23.20	9.00	20.00	26.00	35.00	277.00	49.00

**Table 3:** The optimal hyperparameters for each classifier.

Experiment	Classifier	Hyperparameter	Values	Validation accuracy
Experiment 1	SVM	Cost	5	85.90%
		Gamma	1	
		Kernel	Linear	
	LR	Cost	1	85.90%
		Penalty	L1	
		Solver	Saga	
	Adaboost	N_estimators	80	84.61%
		Learning_rate	0.1	

Experiment 2	SVM	Cost	5	87.49%
		Gamma	0.1	
		Kernel	RBF	
	LR	Cost	3	87.77%
		Penalty	L2	
		Solver	Newton-cg	
	Adaboost	N_estimators	100	86.06%
		Learning_rate	0.1	

**Table 4:** Classifiers testing accuracy, precision, and recall using the optimal hyperparameters.

Experiment	Classifier	Test accuracy	Test precision	Test recall
Experiment 1	SVM	93.28%	93.42%	94.67%
	LR	91.04%	89.87%	94.67%
	Adaboost	91.79%	93.24%	92.00%
	Voting	94.03%	93.51%	96.00%

Experiment 2	SVM	91.79%	92.11%	93.33%
	LR	93.28%	93.42%	94.67%
	Adaboost	89.55%	94.20%	86.67%
	Voting	93.28%	93.42%	94.67%

**Table 5:** Comparison of the results using forward feature selection.

Features	Classifier	Number of features	Features selected	Test accuracy
Experiment 1				
Forward selection	SVM	15	{Sex, age, MCHC, RDW, platelet count, HGB, HCT, NEU%, LYMPH%, BASO#, NEU#, MONO#, chloride, anion gap, SGPT}	89.55%
	LR	30	{Sex, age, MCV, MCHC, RDW, platelet count, MPV, HGB, HCT, WBC, RBC, MONO%, EOS%, NEU%, LYMPH%, BASO%, BASO#, sodium, NEU#, LYMPH#, MONO#, EOS#, potassium, chloride, CO2, anion gap, GGTP, ALP, SGOT, SGPT}	91.04%
	Adaboost	19	{Sex, age, MCV, platelet count, MPV, RBC, MONO%, EOS%, NEU%, BASO%, sodium, LYMPH#, EOS#, potassium, chloride, anion gap, GGTP, SGOT, SGPT}	88.81%
	Voting	30	{Sex, age, MCH, MCV, MCHC, RDW, platelet count, MPV, HGB, HCT, WBC, RBC, MONO%, EOS%, NEU%, LYMPH%, BASO%, BASO#, sodium, NEU#, LYMPH#, MONO#, EOS#, potassium, chloride, CO2, anion gap, GGTP, ALP, SGOT}	94.03%

Experiment 2				
Forward selection	SVM	16	{Sex, age, platelet count, MPV, HCT, EOS%, NEU%, LYMPH%, BASO%, BASO#, sodium, NEU#, EOS#, potassium, chloride, SGOT}	88.81%
	LR	20	{Sex, age, MCHC, RDW, platelet count, MPV, HGB, HCT, WBC, RBC, BASO%, SODIUM, NEU#, MONO#, potassium, CO2, anion gap, GGTP, ALP, SGPT}	93.28%
	Adaboost	6	{Sex, age, MPV, HGB, MONO%, BASO#}	85.82%
	Voting	29	{Sex, age, MCH, MCV, MCHC, RDW, platelet count, HGB, HCT, WBC, RBC, MONO%, EOS%, NEU%, LYMPH%, BASO%, BASO#, SODIUM, NEU#, MONO#, EOS#, potassium, chloride, CO2, anion gap, GGTP, ALP, SGOT, SGPT}	91.04%

**Table 6:** Comparison of the results using backward feature selection.

Features	Classifier	Number of features	Features selected	Test accuracy
Experiment 1				
Backward elimination	SVM	16	{Sex, age, MCV, platelet count, MPV, WBC, EOS%, NEU%, LYMPH%, BASO#, SODIUM, EOS#, potassium, chloride, CO2, SGPT}	92.54%
	LR	31	{Sex, age, MCH, MCV, MCHC, RDW, platelet count, MPV, HGB, HCT, WBC, RBC, MONO%, EOS%, NEU%, LYMPH%, BASO%, BASO#, sodium, NEU#, LYMPH#, MONO#, EOS#, potassium, chloride, CO2, anion gap, GGTP, ALP, SGOT, SGPT}	91.04%
	Adaboost	9	{Sex, age, MCHC, RDW, platelet count, MPV, NEU%, potassium, SGPT}	91.04%
	Voting	12	{Sex, age, MCHC, RDW, platelet count, MPV, WBC, MONO%, NEU%, BASO#, potassium, GGTP}	93.28%

Experiment 2				
Backward elimination	SVM	22	{Sex, age, MCH, MCV, MCHC, platelet count, MPV, HGB, HCT, RBC, MONO%, EOS%, NEU%, LYMPH%, BASO%, BASO#, sodium, NEU#, potassium, chloride, anion gap, SGPT}	91.79%
	LR	24	{Sex, age, MCH, MCV, MCHC, RDW, platelet count, MPV, HGB, HCT, WBC, RBC, MONO%, EOS%, NEU%, BASO%, BASO#, sodium, MONO#, potassium, CO2, anion gap, GGTP, SGOT}	92.54%
	Adaboost	6	{Sex, age, platelet count, MPV, NEU%, potassium}	92.54%
	Voting	22	{Sex, age, MCH, MCV, MCHC, RDW, platelet count, MPV, HGB, HCT, WBC, RBC, MONO%, EOS%, NEU%, BASO#, sodium, NEU#, LYMPH#, potassium, chloride, ALP}	92.54%

**Table 7:** Final results of the best-selected classifiers.

Sampling	Classifier	Test accuracy	Test precision	Test recall
Without sampling	SVM	92.54%	92.21%	94.67%
With sampling	LR	93.28%	93.42%	94.67%
With sampling	Adaboost	92.54%	95.77%	90.67%
Without sampling	Voting	94.03%	93.51%	96.00%

## Data Availability

The rheumatoid disease clinical data used to support the findings of this study are available from the corresponding author upon request.
